The article "Padded Dressing with Lidocaine HCL for Reducing Pain during Intravenous Cannulation in Adult Patients: A Randomized Controlled Clinical Trial" was published in 2022. Journal: Biomed Res Int.

# Padded Dressing with Lidocaine HCL for Reducing Pain during Intravenous Cannulation in Adult Patients: A Randomized Controlled Clinical Trial

**DOI:** 10.1155/2022/6128557

**Published:** 2022-04-23

**Authors:** Fatma Ferda Kartufan

**Affiliations:** Department of Anesthesia and Reanimation, Medistanbul Hospital, Istanbul, Turkey

## Abstract

**Objective:**

In this study, we aimed to evaluate the effect of administering lidocaine as a local anesthetic at the puncture site prior cannulation on reduction of pain during intravenous cannulation (IVC).

**Methods:**

A total of 77 patients were divided into two groups as the patients who received a local anesthetic prior IVC procedure (*n* = 40) and the control group (*n* = 37). Patients' demographic data, including age, gender, height, weight and body mass index, IV gauge, IV site, heart rate (HR), and oxygen saturation (SpO_2_) were recorded and analyzed. Patients in both groups scored the pain they felt during IVC through the visual analog scale (VAS) and the verbal descriptor scale (VDS).

**Results:**

No statistically significant difference was found between the two groups in terms of the demographic features. There was no significant difference between the two groups in terms of the cannula gauges and site of IVC. The mean post-IVC HR value was statistically significantly higher compared to pre-IVC in the control group (*p* = 0.032), while no difference was found between the mean pre- and postprocedure HR in the lidocaine group. The mean VAS score was significantly lower in the lidocaine group compared to the control group (*p* < 0.001). There was a significant difference between the groups in terms of the current VDSs. The rate of the patients reporting mild pain was statistically significantly higher in the lidocaine group compared to the control subjects (*p* < 0.001).

**Conclusion:**

According to the results of this study, lidocaine HCL-impregnated padded dressing prior IV cannulation significantly reduced pain sensation during IVC.

## 1. Introduction

Intravenous cannulation (IVC) is the most widely performed invasive procedure in hospitals with up to 70% of hospitalized patients requiring IVC during their stay. Inserting a cannula into a vein is a routinely performed procedure, especially in children. However, this procedure is inconsistently applied in adult patients. IVC is an experience reported by adults as painful [1]. In the cohort studies conducted with adults in different countries (*n* = 712 patients), more than 50% of the respondents had six or more IVCs in the previous 5 years and described the IVC insertion experience as moderately painful or greater on a scale of 0-10 points [2].

Although IVC is less painful compared to many other procedures performed in hospitals, it is a procedure which causes discomfort to patients who are already in a stressful state. Professional and accreditation standards implemented in order to increase quality of service delivered at healthcare institutions underline that pain due to i.v. cannulation should be reduced [3–5]. In a survey of physicians from 71 hospitals, 35% of the participants stated that they occasionally administered a local anesthetic with lidocaine being mostly used before intravenous cannulation [6]. The participants reported the reasons for not administering local anesthetic before cannulation as time wasting by 45%, a lacking indication/need by 35%, and the worry that intravenous cannulation may be more difficult after administering local anesthetic by 21% [6].

Inadequate pain relief is troublesome for the patient and may increase anxiety about future treatment and may prevent the patient to seek medical help in future health-related problems [7]. Furthermore, fear of the IVC can trigger an automatic response, leading to vasoconstriction [8]. This in turn makes the cannulation process difficult, may require several attempts to achieve access, and thus increases the risk of infection and other complications [9].

So far, several methods have been used to reduce IVC pain, including local anesthetic injection, topical anesthetic, ice application, and valsalva maneuver [10]. However, none of these methods exhibited a clear superiority over the others. There is no clear consensus about which method is the best option to relieve pain induced by IVC. Jeong and Yoon reported that local warming of the intravenous access site by 43°C forced air for 1 minute is slightly more effective in reducing propofol injection pain compared to preadministration of lidocaine [11]. Datema et al. used lidocaine spray as a local analgesic for intravenous cannulation and reported that local administration of lidocaine was not effective in reducing pain during i.v. cannulation [12]. Application of spray cooling agents on the puncture site provide some temporary anesthesia at the cannulation site. However, inconsistent results have been reported regarding this application [2]. The objective of this study was to evaluate the effect of administering local anesthetic (lidocaine) at the IVC site prior cannulation on pain relief.

## 2. Material and Methods

### 2.1. Patients

This study was designed as a clinical prospective, randomized controlled, double-blind study. Before the beginning, the study protocol was approved by the local ethics committee of our hospital with the 09/09/2018 dated and 883 numbered decision. All patients were informed regarding the objectives of the study and gave verbal and informed written consent. The study was performed following the ethics principles of the 1964 Declaration of Helsinki (DoH) and its later amendments.

A total of 77 patients, aged 23-79 years, who presented to our hospital and underwent intravenous cannulation for various reasons were included in this study. Patients aged under 18 years or over 80 years, who did not give informed consent for participation, those needed urgent IVC for emergency procedures, patients with allergy to amide group local anesthetics or their ingredients, and those with any pathology at puncture site and skin disease were excluded from the study. In addition, patients with vagal stimulation, fever, fluid deficiency, malignancy, those receiving chemotherapy, and patients with failed padding were also excluded. Patients were divided into two groups as the patients who received a local anesthetic prior IVC procedure (*n* = 40) and the control group without any application before the cannulation (*n* = 37). The groups consisted of volunteer patients and were created through randomization. The randomization was carried out with a computer using the Research Randomizer statistical software (http://www.randomizer.org). Flowchart of the study is shown in Figure 1.

Patients' demographic data, including age, gender, height, weight and body mass index, gauge of the canula, and IVC site were obtained from the patient files. Pre- and postprocedure vitals: heart rate (HR) and oxygen saturation (SpO_2_) were recorded during procedure by ward nurses via “Nellcor portable SpO_2_ patient monitoring system-PM10N, COVIDIEN, and ABD and analyzed from recordings. Patients in both groups scored the pain they felt during IVC through the visual analog scale (VAS) and the verbal descriptor scale (VDS) right after manipulation. In addition, patients in both groups also scored their pain during their previous IVC experience again through VDS.

### 2.2. Procedure

In the control group; a 10 mL 0.9% isotonic sterile liquid-impregnated padded dressing was adhered to the skin where IVC was planned and left for 15 minutes. The IVC was then performed. In the treatment group, a padded dressing impregnated with lidocaine HCL (Vemcaine© 10% pump spray solution, VEM Ilac Sanayi ve Tic. A.S., Istanbul, Türkiye) was adhered to the skin where IVC was planned and left for 15 minutes. The IVC was then performed. Nurses in the research who performed the padded dressing and IVC and those who collected the VAS scores were blinded to the study. Data obtained were statistically analyzed and compared between the two groups.

### 2.3. Statistical Analysis

The power analysis of the study was completed through the GPower (Version 3.1.9.2) package program. The effect size of the study was calculated as 0.53. Accordingly, using an effect size of 0.53, the power of the study with 37 patients in the treatment group and 40 control subjects was found as 82.8% at a significance level of 0.05.

Statistical analysis of the data obtained in this study was performed utilizing the SPSS version 26.0 (SPSS, Statistical Package for Social Sciences, IBM Inc., IL, USA). Numerical variables are expressed with descriptive statistics (mean ± standard deviation), while categorical variables are given as frequencies (number, percentage).

Normality of the numerical variables was tested with the Kolmogorov-Smirnov method, and the variables were found to be normally distributed. Therefore, parametric statistical methods were used in the analysis. *p* < 0.05 values were considered statistically significant.

## 3. Results

A total of 77 volunteer patients were included in this prospective study with 37 being in the lidocaine group and 40 in the control group. The mean age of the patients was 39.22 ± 11.72 years in the lidocaine group and 39.33 ± 11.43 years in the control group with no statistically significant difference between them (*p* = 0.967). Of the patients in the lidocaine group, 17 (45.9%) were female and 20 (54.1%) were male, while these figures were 21 (52.5%) and 19 (47.5%), respectively, in the control group. No statistically significant difference was found between the two groups in terms of gender (*p* = 0.565). Demographic characteristics of the patients are given in Table 1.

Looking at the IV gauges, 20 (54.1%) patients received 20 gauge (0.9 mm), and 17 (45.9%) patients received 22 gauge (0.7 mm) IV cannulation in the lidocaine group. Nineteen (47.5%) patients received 20 gauge (0.9 mm), and 21 (52.5%) patients received 22 gauge (0.7 mm) IV cannulation in the control group. There was no statistically significant difference between the lidocaine and control groups in terms of the IV gauges (Chi − square = 0.330; *p* = 0.565).

IVC cannulation was established in the dorsum of the hand (DOH) or the antecubital fossa in all patients. No statistically significant difference was found between the two groups in terms of the cannulation sites (Chi − square = 0.275; *p* = 0.600). Cannulation sites according to the groups are shown in Figure 2. All 77 IVC managements were successfull at the first attempt. No adverse effect was observed in both groups following IVC.

The mean heart rate (HR) and oxygen saturation (SpO_2_) values of both groups were recorded pre- and postprocedure and compared both between the groups and within the groups themselves. Accordingly, the mean pre-IVC SpO_2_ value was statistically significantly lower in the lidocaine group compared to the controls (97.59 vs. 98.18; *p* = 0.025). In addition, pre-IVC SpO_2_ value was statistically significantly lower in the lidocaine group compared to post-IVC value (97.59 vs. 98.89; *p* < 0.001). The mean post-IVC HR value was statistically significantly higher compared to pre-IVC in the control group (76.43 vs. 74.42; *p* = 0.032) (Table 2).

Pain, which the patients felt during IV cannulation, was evaluated using VAS and VDS scales. Accordingly, the mean VAS score was significantly lower in the lidocaine group compared to the control group (*t* = 10.455; *p* < 0.001). VAS scores of the groups are depicted in Figure 3.

Pain, which the patient felt, was also evaluated with verbal descriptor scale (VDS) in comparison with previous experience. Accordingly, previous VDS was reported as mild pain by 15% and moderate pain by 85% of the patients in the control group, whereas previous VDS was reported as mild pain by 27% and moderate pain by 73% of the patients in the lidocaine group. The current VDS was reported as mild pain by 10% and moderate pain by 90% of the patients in the control group, while the current VDS was reported as mild pain by 91.9% and moderate pain by 8.1% of the patients in the lidocaine group.

As a result of the chi-square analysis, no statistically significant difference was found between the groups in terms of the previous VDS scale, while there was a significant difference between them in terms of the current VDSs. The rate of the patients reporting mild pain was statistically significantly higher in the lidocaine group compared to the control subjects (*p* < 0.05). And thus, the rate of the patients reporting moderate pain was statistically significantly higher in the control group compared to the lidocaine group (*p* < 0.05).

As a result of McNemar analysis, no statistically significant difference was found between the previous and current VDSs in the control group, while there was a significant difference between the previous and current VDSs in the lidocaine group. Accordingly, the rate of the patients reporting mild pain was statistically significantly higher with the current VDS than the previous VDS (Table 3).

## 4. Discussion

In this study, we investigated whether the application of lidocaine HCL-impregnated padded dressing prior IV cannulation could reduce pain. Our findings give the answer absolutely “YES” to this question.

In our study, demographic characteristics (age, gender, and BMI) of the lidocaine and control groups were statistically similar. Likewise, in a study by Aygun et al. comparing ice and lidocaine-prilocaine cream mixture in the reduction of pain during IVC, age, and gender were similar between the groups [10]. In another study by Page and Taylor, age and gender were similar between the patients receiving vapocoolant spray and those receiving subcutaneous lidocaine injection prior IVC for pain relief [13]. Our findings are consistent with the literature in terms of the demographic features.

The gauge of the cannulae ranged between 16 and 23 in the literature [1]. In a survey study with 178 physicians, it was reported that all the anaesthetists used local anaesthetic when inserting a cannula larger than 18 gauge [14]. In the present study, we used 20 Gauge IV cannulae in 39 and 22 Gauge cannulae in 38 patients in total. There was no significant difference between the groups in terms of the IVC gauges (*p* = 0.565). Twenty gauge (0.9 mm) cannulae were also used in the studies by Burke et al., Ganter-Ritz et al., and Goudra et al. [15–17]. In the present study, we did not evaluate the effect of IVC gauge on pain. However, it was reported in a study by van Loon et al. that inserting a smaller-sized peripheral IVC does not result in a lower pain sensation [18].

Factors affecting the site selection for IVC include general condition of the vein, types of drugs to be administered, duration of planned therapy, and size of the cannula versus size of the vein [19]. van Loon et al. proposed that site of cannulation on the extremity is one of the factors significantly associated with pain during IVC [18]. The antecubital fossa and dorsum of the hand (DOH) are the commonly preferred sites for IV cannulation [20]. Since the innervation density of the skin varies depending on the site, pain at various sites is likely to differ [15]. In the present study, we performed IVC in the antecubital fossa in 23 patients and in the DOH in 54 patients in total. There was no statistically significant difference between the groups in terms of the cannulation sites, although we did not analyze the effect of IVC site on pain. Goudra et al. recommended that the antecubital fossa should be the site of choice in the absence of contraindications [17]. Lavery and Smith also reported that the antecubital fossa site has less pain during cannulation than other sites [20].

Studies have reported that painful stimuli like IVC insertion can cause an autonomic nervous system response that increases a patient's heart rate (HR) [22, 23]. Therefore, some clinicians use HR to evaluate pain in their patients. In our study, HR of the groups was evaluated with the dependent samples *t* test. Accordingly, postprocedure HR was statistically significantly higher compared to preprocedure HR in the control group, suggesting that these patients experienced pain during IVC. In fact, no significant difference was found in the lidocaine group, supporting this situation. However, there are studies reporting no effect of pain on HR. In a study by Bartfield et al., changes in HR were not found to be correlated with pain and anxiety associated with IVC [24]. The difference between the results may be attributed to patient selection criteria and the use of local anesthetics prior IVC.

First described in 1921, visual analog scale (VAS) is a psychometric response scale used to measure subjective characteristics and attitudes and has been used for a multitude of disorders as well as medical conditions including pain [25]. VAS is the most commonly used pain scale. Patients are asked to mark the pain they feel on a 100 mm length ruler involving points from 0 to 10, where 0 indicates “no pain” and 10 means “the worst pain possible.” In the present study, VAS was used as a subjective tool to evaluate pain during IVC. In our study, the mean VAS score was significantly lower in the lidocaine group compared to the control group (*p* < 0.001). Lidocaine has been used with different forms of application in numerous studies for pain relief during IVC, but the results reported are controversial. Datema et al. used lidocaine spray (Xylocaine 10% pump spray) and reported that local administration of lidocaine is not effective in reducing pain during IV cannulation. The authors found no significant difference between the lidocaine and placebo spray groups [12]. In a systematic review and meta-analysis network of 27 studies, Bond et al. reported that 1% lidocaine injection was less painful compared to unattenuated IVC. With the lidocaine injection prior IVC, VAS score was -12.97 points less painful compared to the other applications on a 100 mm VAS scale [1]. Bamgbade reported that VAS score was significantly lower with ice application at the puncture site compared to lidocaine-prilocaine and control groups [8]. In that study, the mean VAS score was found as 4.1 ± 1.8in the lidocaine-prilocaine group, while the mean VAS value was found as only 2.62 in the lidocaine group in our study. As stated above, lidocaine was used in the form of injection, infiltration, or spray in the previous studies. In our study, we tried a novel method with lidocaine HCL-impregnated padded dressing used to reduce pain during IVC, and successful results were obtained as evidenced by VAS scores.

The verbal descriptor scale (VDS) is a series of descriptive statements that refer to different levels of pain severity or intensity. In the VDS, patients select the phrase that best describes their current pain. In our study, we used mild and moderate pain statements, because there was no patient reporting severe pain. Whereas there was no significant difference between the previous and current VDSs in the control group, mild pain was significantly commonly reported by the patients in the lidocaine group for the current VDS compared to the previous VDSs (*p* < 0.001), indicating that pain felt during IVC significantly decreased in the lidocaine group. Kahre et al. compared effects of pain relief during IV insertion using bacteriostatic normal saline and 1% buffered lidocaine and found no significant difference between the groups in terms of VDS. However, the authors did not compare the current VDSs with the previous ones [26]. Different applications of lidocaine among studies make a healthy comparison challenging.

### 4.1. Study Limitations

The major limitations of this study are the relatively small number of patients and being conducted in a single center. Therefore, our results cannot be generalized. In addition, the effects of IV gauges and insertion sites could not be assessed. Finally, we could not evaluate SpO2 values because of the small number of patients. SpO2 could be assessed in further larger-scale studies. Lack of a significant difference between the lidocaine and control groups increases the quality of the study. The most important strength of our study was the finding that both VAS and VDS scores significantly improved with the novel form of lidocaine application.

## 5. Conclusion

According to the results of this study, hydrochloride lidocaine HCL-impregnated padded dressing prior IV cannulation significantly reduced pain sensation during IVC. In addition, HR significantly increased in the control group, while HE was not significant between pre- and postprocedure in the lidocaine group, indicating pain relief. Finally, further multicenter studies with a larger series of patients are needed to support our findings.

## Figures and Tables

**Figure 1:** Flowchart of the study.

**Figure 2:** Distribution of the IV cannulation sites according to the groups.

**Figure 3:** Visual analog scale (VAS) scores of the groups.

**Table 1:** Demographic features according to the groups.

	Control (𝑛 =40)		Lidocaine (𝑛 =37)		Chi-square	*p*
	*n*	%	*n*	%		
*Gender*					0.330	0.565
Female	21	52.5	17	45.9		
Male	19	47.5	20	54.1		
	Mean	SD	Mean	SD	*t*	*p*
Age (years)	39.33	11.43	39.22	11.72	0.041	0.967
Height (cm)	172.15	8.96	172.92	9.09	-0.374	0.710
Weight (kg)	71.67	11.33	75.92	14.01	-1.467	0.147
BMI (kg/m^2^)	24.08	2.37	25.32	4.07	-1.651	0.103

*t*: independent sample *t* test.

**Table 2:** Inter- and intragroup comparison of the mean oxygen saturation and heart rate values.

	Control (*n* = 40)		Lidocaine (*n* = 37)		*t*	*p*
	Mean	SD	Mean	SD		
SpO_2_ 1	98.18	0.98	97.59	1.24	2.289	*0.025* ^∗^
SpO_2_ 2	98.63	1.63	98.89	1.26	-0.799	0.427
	*t* ^b^ = −1.461 *p* = 0.152		*t* ^b^ = −6.853 *p* = 0.0001^∗^			
HR 1	74.42	11.40	74.54	8.62	-0.050	0.960
HR 2	76.43	11.53	76.27	9.49	0.064	0.949
	*t* ^b^ = −2.224 *p* = 0.032^∗^		*t* ^b^ = −1.599 *p* = 0.119			

*t* ^a^: independent sample *t* test (intergroup differences); *t*^b^: dependent sample *t* test (intragroup differences); ^∗^*p* < 0.05.

**Table 3:** Comparison of the previous and current VDSs between and within the groups.

	Control (*n* = 40)		Lidocaine (*n* = 37)		Chi-square	*p*
	*n*	%	*n*	%		
*Previous VDS*					1.689	0.194
Mild pain	6	15.0	10	27.0		
Moderate pain	34	85.0	27	73.0		
*Current VDS*					51.569	*0.0001* ^∗^
Mild pain	4	*10.0*	34	*91.9*		
Moderate pain	36	*90.0*	3	*8.1*		
Mc Nemar	0.625		*0.0001* ^∗^			

^∗^ *p* <0.05.

## Data Availability

Data used in this study are included in the manuscript.
